The article "Glymphatic System: Emerging Therapeutic Target for Neurological Diseases" was retracted in 2023. Reasons: suspected computer-generated content; unreliable results or conclusions; concerns about the data; concerns about the results or conclusions.

# Glymphatic System: Emerging Therapeutic Target for Neurological Diseases

**DOI:** 10.1155/2022/6189170

**Published:** 2022-06-11

**Authors:** Xianjun Xuan, Guoyi Zhou, Caihong Chen, Anwen Shao, Yunxiang Zhou, Xiaobo Li, Jiaqi Zhou

**Affiliations:** ^1^Department of Neurology, Hangzhou Ninth People's Hospital, Hangzhou, China; ^2^The Fourth School of Clinical Medicine, Zhejiang Chinese Medical University, Hangzhou, China; ^3^Department of Neurosurgery, The Second Affiliated Hospital, School of Medicine, Zhejiang University, Hangzhou, China; ^4^Department of Surgical Oncology, The Second Affiliated Hospital, School of Medicine, Zhejiang University, Hangzhou, China; ^5^State Key Laboratory for Diagnosis and Treatment of Infectious Diseases, National Clinical Research Center for Infectious Diseases, Collaborative Innovation Center for Diagnosis and Treatment of Infectious Diseases, The First Affiliated Hospital, College of Medicine, Zhejiang University, China

## Abstract

The newly discovered glymphatic system acts as pseudolymphatic vessels subserving brain waste clearance and is functionally dependent on astrocytic aquaporin-4 channels. The glymphatic system primarily functions during sleep as an interchange between cerebrospinal fluid and interstitial fluid, with cerebrospinal fluid flowing into the parenchyma via the perivascular spaces and then exchanging with interstitial fluid. The discovery of meningeal lymphatics helps refine the conceptual framework of glymphatic pathway, as certain waste products collected alongside perivascular spaces ultimately drain into the cervical lymph nodes via meningeal lymphatics, whose function regulates the functioning of the glymphatic system. The glymphatic and meningeal lymphatic systems are critical for the homeostasis of central nervous system, and their malfunctions complicate cerebral dysfunction and diseases. The present review will shed light on the structure, regulation, functions, and interrelationships of the glymphatic system and meningeal lymphatics. We will also expound on their impairments and corresponding targeted intervention in neurodegenerative diseases, traumatic brain injury, stroke, and infectious/autoimmune diseases, offering valuable references for future research.

## 1. Introduction

Homeostasis is vital for tissue health. Excess fluid and soluble proteins from the interstitial tissue space are returned to the circulation via the lymphatic system in peripheral tissue and organs [1–3]. Although the central nervous system (CNS) has a high metabolic rate, it lacks a conventional lymphatic system, which has made brain waste clearance, cerebrospinal fluid (CSF)/interstitial fluid (ISF) outflow mechanisms, and neuromonitoring a realm of enigmas and mystery for a long time [2, 4]. Emerging studies have reported the existence of meningeal lymphatics and demonstrated that there is a perivascular pathway acting as pseudolymphatic vessels for brain waste clearance. It functionally depends on aquaporin-4 (AQP4) channels, the main water channels of astrocytes, thereby referred to as a glial-lymphatic or glymphatic system [5–7]. This unravels several questions, casting a spotlight.

CSF and ISF constitute the extracellular fluid of the brain [8]. The former is mainly secreted by the choroid plexus and is considered the leading way to remove metabolic waste products from CNS [5, 9]. However, the latter may be secreted by blood-brain barrier (BBB) and surrounds the brain parenchyma, delivering fluid and solute to brain cells and directly removing waste products from those cells [10–13]. CSF and ISF exchange plays a pivotal role in the waste clearance within CNS, including toxic proteins like amyloid *β* (A*β*) and tau [14]. Notably, the underlying mechanisms of extracellular fluid circulation and metabolism are strongly correlated with the glymphatic system and meningeal lymphatics, significantly affecting the waste clearance and fluid balance. Mechanically, the glymphatic system functions as an interchange between them and facilitates their exchange [6]. Meningeal lymphatics perform the function of CSF absorption and waste clearance, transporting immune cells and soluble substances to peripheral lymph nodes [15–17]. Generally, there are three pathways of CSF drainage: (1) CSF from the subarachnoid space drains directly into the blood via the arachnoid villi of the superior sagittal sinus, (2) CSF from the subarachnoid space drains into the lymph nodes via the subarachnoid spaces around the olfactory nerves and nasal lymphatics, and (3) meningeal lymphatics disgorge macromolecules and immune cells of CSF into the cervical lymph nodes [18–21].

Given their critical impact on the maintenance of CNS homeostasis, the impairments of glymphatic system and meningeal lymphatics may lead to cerebral dysfunction and diseases [8]. Increased evidence has revealed that the dysfunction of glymphatic/meningeal lymphatic system is implicated in various neurological diseases, such as Alzheimer's disease (AD), stroke, traumatic brain injury (TBI), and infectious/autoimmune diseases [21–25]. This study reviews the recent findings concerning characteristics, functions, and relationships of glymphatic system and meningeal lymphatics. We also elaborate on the crosstalk between glymphatic/meningeal lymphatic system and neurological disorders and discuss corresponding targeted interventions, which may lend significant therapeutic promise.

## 2. The Discoveries of Glymphatic and Meningeal Lymphatic Systems

### 2.1. Classical Model of the Circulation of Extracellular Fluid

It is traditionally thought that the choroid plexus secretes CSF. It then flows from lateral ventricles to the third ventricle through the foramen of Monro, subsequently passing across the aqueduct to the fourth ventricle, where CSF enters subarachnoid space through the apertures of Magendie and Luschka and is eventually absorbed into the blood at the arachnoid villi [9, 26]. However, there was no consensus on the mechanism for draining through arachnoid villi. Researchers did not find direct evidence to confirm the function of arachnoid villi [27, 28]. Ma et al. recently proposed that lymphatic outflow was the primary route to draining CSF [29]. In this model, the choroid plexus is the leading site of CSF formation, secreting approximately 80-90% of the total CSF [8, 30]. Unlike BBB, there are no tight junctions between the endothelial cells in the choroid plexus, which is beneficial to fluid infiltration in blood [2, 8]. However, tight junctions are present between epithelial cells to regulate CSF secretion [2, 8, 30]. The main driver of the CSF secretion is metabolic energy to fuel the Na-pump [31]. In addition to the osmotic pressure gradient, the high AQP1 expression at the apical membrane contributes to high fluid permeability [26]. Besides arachnoid villi, CSF absorption can be achieved through two other routes: (1) passing along olfactory nerves across the cribriform plate to the nasal mucosa and then entering the cervical lymphatics or (2) flowing through the spinal nerve root into blood or lymph [10, 32].

Another type of extracellular fluid of the brain, ISF, is produced by the capillary-astrocyte complex of BBB, providing a necessary environment for brain cells [10, 12, 26]. ISF surrounds the brain parenchyma with the metabolic waste products of brain cells dissolved inside and drains to CSF to renew itself, while CSF acts like lymphatics and causes eventual waste removal from CNS [8]. Although CSF's clearance of waste from the brain is widely accepted, it remains unclear how CSF exchanges with ISF to remove metabolic waste products.

### 2.2. Novel Discoveries of the Circulation of Extracellular Fluid

Due to developing neuroanatomy, molecular biology, and neuroimaging, discoveries regarding the circulation of CSF and ISF have emerged. For instance, researchers have found that choroidectomy did not cure hydrocephalus, suggesting the existence of other CSF sources [10, 33]. Correspondingly, novel assumptions have been put forward. Brinker et al. proposed a model in which CSF and ISF are formed and absorbed directly in the capillaries rather than passing through the choroid plexus to arachnoid villi [26]. Nevertheless, this model was inadequate as CSF flow through the aqueduct was observed using magnetic resonance imaging (MRI) [34]. Some researchers combined the two abovementioned models to generate a new one, which was thought to provide new insights into CSF formation [2]. More attractively, recent work has demonstrated the presence of glymphatic and meningeal lymphatic systems, uncovering more precise mechanisms underlying the exchange and outflow of extracellular fluid.

### 2.3. The Discovery of the Glymphatic System

Recent discoveries about the brain's glymphatic system have garnered considerable debate [6, 17, 35]. Many details about glymphatic systems were described decades ago. For instance, Cserr et al. conducted several experimental studies by injecting traceable solutes into the brain to identify the pathway of fluid removal [36–38]. They also found that removal rates of traceable solutes were almost identical, regardless of the molecular size and weight [37, 38]. It was concluded that the communication of ISF and CSF occurred in a specialized pathway in the brain by convection [14]. Moreover, studies revealed that CSF could penetrate the brain parenchyma through perivascular space via convection [8, 39, 40]. However, this conclusion was questioned for decades before Iliff et al. made a breakthrough in 2012 [6, 14]. Iliff et al. used two-photon imaging and Tie2-GFP: NG2-DsRed double reporter mice to investigate the flow of CSF in the brain parenchyma [6]. They demonstrated CSF and ISF exchange and the efflux of mixed CSF and ISF out of the brain and the perivenous space.

Given that the function of this perivascular pathway was similar to that of the lymphatic system, with astrocytic AQP4 playing a crucial role in it, it was therefore termed the glial-lymphatic system or glymphatic system [6]. Notably, Carare et al. concluded that solutes drained out along the basement membranes of capillaries and arteries, flowing in the direction opposite to arterial blood [18]. The outflow pathway of glymphatic system remains a debate. Bakker et al. proposed that the existence of these two pathways, separated by meningeal sheets, could explain the debate [41]. They also proposed that different research methods might contribute to different findings [41]. However, this debate is yet to be settled by experiments.

The glymphatic system consists of periarterial CSF, flowing in the same direction as blood, propelled by the pulsatility of the arterial wall [42, 43]. CSF and ISF mix in a process aided by AQP4 water channels abundant at the vascular astrocytic end-feet [44]. The influx of fluid across BBB or extrachoroidal sources of CSF may also contribute to glymphatic flow [45–47]. CSF and ISF mixture leaves the brain via the perivenous space and along cranial and spinal nerves. This fluid is eventually transported out of CNS by traditional lymphatic vessels located in the meninges and the soft tissue surrounding the skull. The current wave of great interest in the glymphatic system is probably that the glymphatic system concept has articulated a function of the transport system by demonstrating its role in A*β* clearance [6]. The glymphatic system clears key proteins involved in neurodegeneration. In contrast, inhibiting glymphatic system transport accelerates protein accumulation and cognitive decline in mouse models of Alzheimer's disease, traumatic brain injury, and Parkinson's disease [20, 25, 48], indicating that the glymphatic system is an attractive brain waste removal system.

### 2.4. The Discovery of Meningeal Lymphatics

In the 18th century, physician Paolo Mascagni discovered lymphatic vessels in the meninges and made people conscious of their existence [32]. However, his view was not initially understood and accepted by others [32]. Over the next 200 years, several studies suggesting the presence of lymphatic vessels in the meninges [49–51] appeared with questions [32]. Researchers recently confirmed Paolo's conjecture by detecting the lymphatic epithelial cell markers (e.g., LYVE-1, VEGFR3, PDPN, CCL21, and PROX1) in mouse meningeal vessels using immunofluorescence staining [15, 17]. Alitalo et al. addressed the existence of meningeal lymphatic vessels in CNS alongside the arteries, veins, and cranial nerves in mice [15]. It was further discovered that meningeal lymphatics exist not only in mice but also in other animals and humans [16, 32] (Table 1). Zhou et al. visualized the clearance of meningeal lymphatics based on brain 3-dimensional T1-weighted imaging in humans, which supported the existence of meningeal lymphatic vessels in the human CNS [52]. Furthermore, Louveau et al. showed that the characteristics of meningeal lymphatics are consistent with the initial lymphatic vessels, both lacking smooth muscle cells [17].

The brain was considered immune-privileged because of the absence of a lymphatic system in CNS [53]. The concept of CNS immune privilege was proposed for allografts surviving longer in the brain compared with the periphery [54]. Another experiment showed that skin allografts into the brain caused late graft rejection, consistent with the findings mentioned above [55]. However, recent evidence has overturned the idea that CNS lacks lymphatic vessels [16, 35]. The discovery of meningeal system makes CNS connected to peripheral lymphatics [54]. As discussed above, CSF drained antigens, activated T cells and other immune cells to cervical lymph nodes through the meningeal system, and then induced an immune response in cervical lymph nodes [4, 17, 54]. This may explain why allografts survived longer in the brain [4].

The meningeal system played a key role in immune surveillance. The immune cells and antigen-presenting cells (APCs) in CSF were drained to cervical lymph nodes via the meningeal system [54]. Antigens from the brain presented to the APCs activate immune cells such as T cells in lymph nodes and induce them to enter the brain across BBB using specific adhesins (ICAM-1 and VCAM-1) [54]. In addition, lymphatic endothelial cells of meningeal vessels contribute to the tolerance of T cells in CNS, which is vital in maintaining the homeostasis of CNS [53].

## 3. Glymphatic System and Meningeal Lymphatics

### 3.1. AQP4 in the Glymphatic System

#### 3.1.1. The Distribution of AQP4

AQP4 is one of 14 aquaporins that are only found on astrocytes and are primarily found in their foot processes [10, 56, 57]. AQP4 is expressed as a tetramer [8]. There are two isoforms of AQP4, M1, and M23 [56]. The supramolecular structure assembled by M23 is called orthogonal arrays of particles (OAPs), which can enhance water permeability and promote the polarization of AQP4 to the astrocyte end-feet. Astrocytes stretch these particles to the microvessels to constitute the perivascular space and glial limiting membranes and sheathe the BBB [56, 57]. Moreover, AQP4 anchors to the dystrophin-associated protein complex (DAPC) attached to the perivascular glial basement membrane [8]. These characteristics reflect the high density of AQP4 in the perivascular space.

#### 3.1.2. The Function of AQP4

AQP4 is a regulator for the transcellular transport of water and facilitates the rapid movement of water flow across the membrane [58]. The high AQP4 expression in perivascular space plays a vital role in the influx and efflux of the glymphatic pathway [6]. AQP4 reduces the resistance of CSF and ISF exchange in the glymphatic system [4, 6]. Iliff et al. found that the flow velocity of tracer solutes did not reduce in the periarterial space but significantly reduced when passing from the perivascular space to the interstitial space in AQP4-null mice, suggesting that AQP4 affects the fluid flow in this interface [6]. Additionally, the removal rates of interstitial solutes and A*β* were reduced by 70% and 55%, implying that AQP4 is critical for the clearance of brain waste products [6]. These findings are consistent with other studies, revealing that the function of the glymphatic system mainly depends on AQP4 [59, 60].

### 3.2. The Driving Force of the Glymphatic System

#### 3.2.1. The Driving Force

The fluid transportation of glymphatic system involves multiple mechanisms [8]. Iliff et al. showed that ligation of the internal carotid artery reduced CSF influx while dopamine, an inotropic adrenergic agonist, increased it [42]. They suggested that cerebral arterial pulsation, including its amplitude and frequency, was a primary driving force for CSF influx in the glymphatic system [42]. This conclusion is further verified by Liu et al., who found that acute alcohol exposure reduced cerebral vascular pulsation, provoking the reduction of CSF influx in the glymphatic system [61]. Furthermore, the respiratory-related pulsatile cycle promotes the centripetal venous fluid flow, augmenting perivenous spaces and driving CSF outflow in the glymphatic system [62].

Intracranial pressure (ICP) is another driving force of the glymphatic system [58]. When CSF communicates with the outside, ICP decreases, and the solute clearance rate in the glymphatic system decreases significantly [58]. Meanwhile, ICP is related to the head posture, as it decreases when the head moves from supine to upright [58].

#### 3.2.2. Action Time

The glymphatic system functioning is primarily active during sleep and is primarily suppressed during the awake state [8, 58]. CSF influx can be reduced by 95%, and A*β* clearance can be slowed by half on awakening [63]. Xie et al. suggested that the state of consciousness determined the rate of solute clearance in the glymphatic system in mice rather than the circadian rhythm [63]. They also found that CSF influx increased after inhibiting the adrenergic signaling during wakefulness [63]. Consistent with this, another study found that the glymphatic transport increased by 32% in rats anesthetized with dexmedetomidine, which lowers norepinephrine, plus low-dose isoflurane, which does not, compared with high-dose isoflurane only [64]. Adrenergic signaling activation in the awake state may affect the glymphatic pathway transport.

### 3.3. The Function of the Glymphatic System

As mentioned above, the glymphatic system is an interchange between CSF and ISF and facilitates their exchange to promote waste removal (Figure 1) [4, 6]. As a result, one of the most significant functions of glymphatic system is removing the metabolic waste products [8], which include A*β* and tau and are associated with neurological diseases when accumulated from CNS [65]. The glymphatic system achieves the clearance of lactate from wakefulness to sleep [66].

The glymphatic system also serves as a key player in nutrient distribution [8], brain energy supply (via glucose delivery) [67], and lipid transport and signaling [68]. The diffusion of lipids in the glymphatic system is highly selective, which may be related to the high density of astrocyte-secreted lipoproteins and lipid transport carriers. In contrast, an impaired glymphatic system leads to unselective diffusion of lipid and abnormal astrocyte calcium signaling [68]. The glymphatic system can also facilitate the distribution of apolipoprotein E (ApoE) in the brain, which removes excess A*β* and maintains brain homeostasis [2, 7]. Recent work found that fluid stress opened N-methyl-D-aspartic acid (NMDA) receptors in astrocytes, increasing calcium current, suggesting that the glymphatic system might play a role in mechanotransduction [8].

### 3.4. The Function of Meningeal Lymphatic System and Its Interaction with the Glymphatic System

The novel discovery of meningeal lymphatics as a complementary route for CSF and ISF clearance has attracted much attention [15, 17]. Alitalo et al. disclosed that meningeal lymphatics absorbed CSF from subarachnoid space and brain ISF via the glymphatic system, draining CSF directly into the deep cervical lymph nodes (dCLNs) in mice [15]. Their findings are consistent with those of Zhou et al. [52]. Notably, meningeal lymphatics played a crucial role in the clearance of macromolecules, whose clearance from CNS and transfer from the subarachnoid space into dCLNs could be attenuated and abrogated upon the aplasia of the meningeal lymphatic system [15]. After injecting Evans blue, Louveau et al. found that Evans blue appeared successively in meningeal lymphatics, dCLNs, and superficial cervical lymph nodes (sCLNs) in human samples and mice [17]. They concluded that meningeal lymphatics were the main pathway for draining specific solutes from CSF and ISF into dCLNs [4, 17]. However, Ma et al. declared perineural pathways to be a major route to drain solutes from the brain to dCLNs, as they found that P40D680, a kind of pegylated near-infrared tracers, drained along the perineural (e.g., olfactory nerve and optic nerve) pathway, while no signal was detected in the meningeal lymphatic vessels [29]. These contradictory findings may be explained by the different tracers used, warranting further experiments to uncover the mystery.

CSF delivers cytokines, neurotransmitters, and hormones throughout the brain and removes metabolic waste products away from the brain parenchyma by exchanging with ISF via the glymphatic system [5, 6, 9, 53]. CSF is enriched with interstitial solutes and drains to the periphery mostly through meningeal lymphatics, which play an important role in macromolecule removal (Figure 2) [15]. Notably, the drainage of meningeal lymphatics is positively related to the CSF influx in the glymphatic system [20]. The glymphatic system functioning is regulated by the function of the meningeal lymphatic system [20]. The glymphatic and meningeal lymphatic systems are coupled in the exchange and circulation of the brain's extracellular fluid. The discovery of meningeal lymphatics helps refine the conceptual framework of the glymphatic pathway.

## 4. Glymphatic Pathway and Neurodegenerative Diseases

### 4.1. Neurodegenerative Diseases

Neurodegenerative diseases, a group of clinical diseases including AD, Parkinson's disease, and others, are characterized by the accumulation of pathological proteins, such as A*β*, tau, and *α*-synuclein [2, 69]. AD is the most common neurodegenerative disease, affecting 10-30% of the population over the age of 65 [70]. AD is characterized as a chronic progressive disease that involves cognitive impairment and neuropsychiatric abnormalities [70], with a global burden of US$ 818 billion in 2015, with a 35% increase over the previous five years [71]. AD is generally in an advanced stage when diagnosed [70]. Patients with different AD forms are often accompanied by dementia [72]. The median survival time for AD patients is approximately 7.1 years, an apparent reduction in life expectancy [70]. AD management mainly relies on pharmacotherapies, including NMDA receptor antagonists (e.g., memantine) and cholinesterase inhibitors (e.g., donepezil, galantamine, and rivastigmine). However, their efficacies are limited to slowing down the progress of cognitive impairment [72]. Therefore, novel therapeutics are urgently required.

### 4.2. Crosstalk between the Glymphatic Pathway and AD

AD is featured with the accumulation of amyloid plaques and neurofibrillary tangles of hyperphosphorylated protein tau [65, 69]. The hyperphosphorylated protein tau is often thought to be produced in the later stage of AD [73], and the accumulation of A*β* is considered the predominant cause of AD [73]. A*β* clearance involves a series of mechanisms, including phagocytosis by myelomonocytes, degradation by astrocytes and neurons, and drainage into the peripheral circulation or lymphatic system via the BBB and glymphatic system [74, 75]. Although the drainage route through BBB into blood is responsible for 75% of A*β* removal, the glymphatic pathway is an indispensable alternative route [32], and the impaired glymphatic system is adequate to yield a decreased clearance rate of A*β* and tau [6, 75, 76]. The aggregation of A*β* can inhibit the function of glymphatic system by constricting blood vessels, resulting in glymphatic influx suppression [77].

Moreover, the circulation of A*β* in the brain is mediated by the glymphatic system, and prolonged circulation of A*β* that has not been cleared in time may trigger the formation of amyloid plaques, which reduce the perivascular space of the glymphatic system, impairing the exchange efficiency of CSF and ISF [77]. In addition, amyloid plaques can lead to cerebral amyloid angiopathy (CAA) development [78, 79]. CAA boosts arteriosclerosis and reduces arterial pulsation [78, 79], which in turn further reduces the clearance efficiency of glymphatic system [75]. These discoveries suggest a vicious cycle in which A*β* accumulation facilitates the dysfunction of glymphatic system, resulting in further reduced clearance of A*β* and amyloid plaque formation [75]. The dysfunction of meningeal lymphatics also aggravates AD [20, 80], which is reflected by the critical role meningeal lymphatics play in CSF circulation and macromolecule clearance [4]. Altogether, the impairment of glymphatic/meningeal lymphatic systems may be a risk factor for AD onset and development.

As a determinant of the function of glymphatic system, AQP4 regulates A*β* removal [6, 48]. Iliff et al. found that A*β* clearance decreased by 55% in *AQP4* knockout mice [6]. Similarly, Xu et al. displayed that *AQP4* knockout aggravated A*β* accumulation and the cognitive impairment of A*β* precursor protein/presenilin 1 mice, a pathological model of AD [48]. They also found that *AQP4* knockout did not affect A*β* formation and degradation [48]. Amyloid plaque deposition is mainly associated with the impairment of A*β* clearance rather than the increase of A*β* formation [58]. Moreover, aging is a significant predisposing factor for AD [81]. Although AQP4 expression can increase in the aging brain, the loss of perivascular AQP4 localization increases the vulnerability of the aging brain to the disaggregation of pathological proteins [82]. Zhou et al. demonstrated that the glymphatic system might be impaired in older people, which may accumulate A*β* [52]. Notably, AQP4 and A*β* aggregation also interact, forming a vicious circle. Long-term accumulation of A*β* leads to the atrophy and malfunction of astrocytes, which in turn reduces the clearance of A*β* [48]. Furthermore, amyloid plaque and reactive astrogliosis in AD pathology can inhibit AQP4 polarization to astrocyte end-feet, resulting in a decrease in A*β* removal in the glymphatic system [48, 77].

Sleep deprivation has been revealed to increase AD susceptibility [83–85]. It can induce the impairment of glymphatic system functioning, leading to A*β* accumulation and accelerating amyloid plaque formation [63, 85, 86]. Besides, sleep deprivation-induced glymphatic malfunction hinders ApoE delivery, reducing A*β* clearance across BBB [87]. In addition, sleep deprivation is associated with A*β* production [84]. Shorter sleep time and poor sleep quality can lead to higher levels of A*β* burden [84]. Although we have explained that reduced A*β* clearance mainly accounts for AD occurrence and development [58], we cannot rule out the role of increased A*β* production in AD pathogenesis, which requires further investigation.

### 4.3. Glymphatic Pathway as a Novel Therapeutic Target for AD

The discovery of the glymphatic pathway provides promising strategies for treating AD [80]. The restoration of cerebral arterial pulsation in AD patients can preserve the driving force of the glymphatic system, holding a therapeutic potential [42, 75]. It is suggested that protecting smooth muscle cells to maintain pulsation may prevent AD [75, 88]. AQP4 polarization destroyed by AD in the astrocyte end-feet serves as a candidate mechanism for intervention. N-3 polyunsaturated fatty acids (PUFAs) have been demonstrated to protect the polarization of AQP4, increase A*β* removal in the glymphatic system, and avoid amyloid plaque formation [89]. Melatonin can improve sleep quality, potentially enhancing the activation of the glymphatic system and increasing A*β* removal [83, 90]. However, melatonin has not been revealed to significantly improve cognitive ability in AD patients [90]. More preclinical and clinical studies regarding the precise mechanisms of glymphatic malfunction in AD and related targeted therapy are required.

## 5. Glymphatic Pathway and Traumatic Brain Injury

### 5.1. Traumatic Brain Injury

TBI is the structural or functional disruption of the brain caused by external forces, which often occurs in soldiers and athletes [91–93]. TBI is now considered a public health crisis and a leading cause of death and disability worldwide [91, 92, 94]. TBI incidence is about 349 per 100000 persons per year, of which mild traumatic brain injury (mTBI) accounts for the majority, with an incidence of around 224 per 100000 persons per year [91, 92]. It is estimated that 50% of individuals would be affected by TBI in their lifetime [91]. TBI is a heterogeneous disease with diverse clinical manifestations, complicating the management strategies [92, 95]. This may be attributed to the complexity of the brain and the secondary injury [96]. So far, few effective TBI therapies have been developed [96–98]. TBI survivors usually suffer from various sequelae, including cerebrovascular disease, cerebral concussion, coma [98], and some chronic complications, such as neurodegenerative diseases [99] and sleep disorders [100, 101]. These sequelae impose a more significant burden on societies, patients, and families than TBI itself [98].

### 5.2. Crosstalk between Glymphatic Pathway and TBI

Growing evidence demonstrates that TBI is a risk factor for tauopathies, including AD, chronic traumatic encephalopathy (CTE), and frontal-temporal dementia (FTD) [102–104]. Tauopathy refers to the formation of neurofibrillary tangles (NFT) composed of hyperphosphorylated tau [105]. Mechanically, the glymphatic system is impaired in TBI, leading to the reduction of tau removal and ultimately aggravating the tauopathy [25].

Brain edema is a frequent manifestation of TBI, altering ICP and suppressing the glymphatic system [106]. After TBI, glial scars characterized by hypertrophic glial fibrillary acidic protein- (GFAP-) positive astrocytes and reactive astrogliosis surround the ipsilateral hemispheres, changing the polarization and localization of AQP4 to affect the clearance of glymphatic system, with the recovery time proportional to the severity of TBI [25, 107]. AQP4 expression may not fully recover after 28 days in severe TBI [93]. These post-TBI changes cause the dysfunction of the glymphatic system, resulting in decreased glymphatic influx and waste removal [2, 25]. TBI impairs the clearance of tau and increases the production of tau, further accumulating interstitial tau [108].

The dysfunctional glymphatic pathway is a key player in post-TBI neuroinflammation, a “double-edged sword” that may be beneficial, increasing debris clearance or harm and accelerating nerve cell death [109]. The increased waste due to the dysfunction of glymphatic system can trigger or enhance inflammatory responses [109]. Moreover, the altered association of meningeal vessels and peripheral lymphatics post-TBI may further lead to inflammatory disequilibrium and worse outcomes [109].

The recently discovered enlarged perivascular space (ePVS) may be a marker of the dysfunction of glymphatic clearance [110]. A positive correlation between sleep deprivation and ePVS has been observed in TBI [111]. Sleep disturbances are prevalent following TBI, particularly in mTBI victims [112]. About 80% of mTBIs are linked to sleep disturbances, in which insomnia is the most common [113], underlying the impairments of glymphatic system post-TBI [63]. Sleep deprivation may trigger or aggravate other complications and sequelae of TBI, including neurodegenerative diseases [112].

### 5.3. Glymphatic Pathway as a Novel Therapeutic Target for TBI

Reactive astrogliosis is implicated in a myriad of pathologic mechanisms of TBI, including the loss of AQP4 polarization [25, 57]. Inhibiting reactive astrogliosis may restore the glymphatic system by keeping AQP4 polarized [25]. Studies have demonstrated the potential of stem cells in TBI treatment, and one of the mechanisms is that stem cells may inhibit the reactive astrogliosis by suppressing inflammatory response [114]. Moreover, recent work disclosed that post-TBI anesthetics increased the uptake of dendrimer nanoparticles enriched with anti-inflammation drugs in glial cells, thus enhancing the efficiency of drugs and leading to better restoration of the function of neuroglia and the glymphatic system [115]. However, this finding was obtained in cell experiments [115] and must be further validated *in vivo*. Furthermore, cisternostomy, a novel surgical procedure, can recover ICP and the function of glymphatic system after TBI [106].

## 6. Glymphatic Pathway and Stroke

### 6.1. Stroke

Stroke, the second leading cause of death and the third leading cause of disability worldwide, can be classified into ischemic stroke and hemorrhagic stroke [116–118]. Stroke affects 13.7 million people every year worldwide, with a global annual cost of US$ 34 million [116, 119]. It is estimated that one in every four adults will experience a stroke during their lifetime [116]. Ischemic stroke accounts for 71% of global strokes [116]. The incidences of ischemic stroke in men and women are approximately 133 and 99 per 100,000 persons, respectively [117]. Hemorrhagic stroke includes subarachnoid hemorrhage (SAH) and intracranial hemorrhage (ICH), the incidences of which are 9.1 and 24.6 per 100,000 persons, respectively [120, 121]. The incidence and mortality of stroke have declined gradually over the past two decades [116, 117, 122]. However, the rate of mortality decline has slowed in recent years and is even increasing [119]. Stroke survivors may never fully recover neurological function [121]. The disability-adjusted life-year (DALY) due to stroke was 113 million in 2013 [117]. Therefore, stroke still poses a significant challenge for society. It is necessary to explore a new therapeutic approach.

### 6.2. Crosstalk between Glymphatic Pathway and Stroke

Studies have demonstrated that stroke impairs the glymphatic system [24, 123, 124]. Ischemic stroke induces the dysfunction 3 h postinjury by reduced vascular pulsation and occlusive perivascular space due to thrombus, while the recanalization of arteries after 24 h can recover the function of the glymphatic system [24]. Regarding SAH, the glymphatic system dysfunction occurs 24 h postonset [24]. The impaired glymphatic system caused by SAH may be correlated with the occlusion by blood clots post SAH in the perivascular space, which affects CSF circulation [123]. Notably, ICH seems not to impair the function of glymphatic system [24]. As a result of the dysfunctional glymphatic system, CSF efflux turns to reduce, rendering ICP elevated, which parallels worse outcome poststroke [125]. In addition, A*β* accumulates poststroke, which accelerates the formation of amyloid plaques, CAA, and even dementia [124]. Dementia is one of the common complications of stroke; about a quarter of patients develop dementia three months after stroke onset [126]. In addition, the reduction of glymphatic system clearance after SAH can lead to delayed cerebral ischemia (DCI), which is associated with SAH prognosis [123].

A recent study by Mestre et al. has been cast in the spotlight and may revise our understanding of poststroke edema [127]. Cerebral edema is a prevalent complication of stroke, and its severity is related to patient outcomes [128]. Unexpectedly, Mestre et al. found that increased CSF influx via the glymphatic system was the leading cause of early stage edema after ischemic stroke [127]. Ischemic spreading depolarization, which contributes to the vasoconstriction of cerebral arteries, could change the pressure gradient, provoke ePVS, and double glymphatic influx [127]. In addition, they demonstrated that AQP4 deletion reduced cerebral edema caused by ischemic stroke [127]. However, AQP4 deletion impairs the clearance function of glymphatic system, which may lead to other complications [6]. Thus, the impact of glymphatic system on ischemia stroke under different stages may require further exploration.

Meningeal lymphatics play a vital role in the outcome of ischemic stroke [129, 130]. In addition to the impaired BBB, meningeal lymphatics represent another pathway for peripheral immune cells, such as T and B cells, to invade brain parenchyma and aggravate the neuroinflammation during ischemic stroke [131, 132]. Mast cells in the meninges may amplify the inflammation response and worsen the prognosis of stroke patients [132]. Moreover, the ingrown meningeal lymphangiogenesis into the injured brain parenchyma post vascular injury can increase the clearance of interstitial fluid to resolve cerebral edema and promote vascular regeneration [130]. Conversely, the hypoplasia of meningeal lymphatics does aggravate the severity of ischemic stroke in transient MACO [129]. Hence, it appears likely that meningeal lymphangiogenesis is linked to the outcome of ischemic stroke [129].

### 6.3. Glymphatic Pathway as a Novel Therapeutic Target for Stroke

Targeting the glymphatic system and meningeal lymphatics has the therapeutic potential for stroke and its complications and sequelae based on the roles mentioned above [129, 130]. Injection of tissue plasminogen activator can dissolve thrombus in vessels or perivascular space to recover the function of glymphatic pathway [24, 133]. The recovery of glymphatic system functioning is beneficial to A*β* clearance, and protein tau, among other interstitial solutes, reduces the incidence of poststroke dementia [124]. Moreover, dexmedetomidine administration holds the promise of reversing the impaired glymphatic system poststroke [133]. In addition, increasing the plasma osmolality has been suggested to subserve the function of glymphatic system by accelerating glymphatic inflow speeds [134]. According to Mestre et al. [127], this may aggravate cerebral edema in the early stage of ischemic stroke, meriting further study.

## 7. Glymphatic Pathway and Infectious or Autoimmune Disease

Besides the diseases mentioned above, the glymphatic pathway is related to diseases, including infectious and autoimmune diseases. Microglia and type I astrocytes, the crucial innate immune cells that reside in CNS, are considered part of the glymphatic pathway [135], accounting for the close relationship between the glymphatic pathway and brain infection/inflammation [53, 135]. Recently, novel coronavirus- (SARS-CoV-2-) infected disease (COVID-19) started spreading worldwide. Lavi and Cong found that microglia and type I astrocytes infected with murine coronavirus (MHV-A 59), whose pathogenesis is similar to that of SARS-CoV-2, released proinflammatory cytokines, such as IL-1, IL-2, IL-6, TNF, and interferons [135], providing valuable insight into the crosstalk of glymphatic pathway and COVID-19.

Multiple sclerosis (MS), characterized by the invasion of auto-reactive T cells, is one of the common autoimmune diseases of CNS [21, 54]. Experimental autoimmune encephalomyelitis (EAE) is the most common animal model to explore the molecular immune in CNS [54]. Louveau et al. demonstrated that ablation of the meningeal lymphatics could prevent the interaction of T cells and APC and the activation of T cells in dCLNs, resulting in the reduced invasion of activated T cells into the brain and ameliorating the EAE [21]. They concluded that meningeal lymphatics played a critical role in the immune surveillance and the inflammatory response regulation of CNS [21]. As a result, meningeal lymphatics may be a therapeutic target for CNS autoimmune disease.

## 8. Conclusion

CSF has always been considered to play a vital role in CNS metabolism. The characterization of glymphatic/meningeal lymphatic system has led to a more nuanced understanding of the exchange and circulation of CSF and ISF in the brain. The glymphatic and meningeal lymphatic systems add to our understanding of metabolic waste drainage and immune privilege. However, more research is required for further understanding of these systems. The function of glymphatic system is linked to different physiological conditions, such as cerebral vascular pulsation, state of consciousness, and body posture, and is partially regulated by meningeal lymphatics. The glymphatic/meningeal lymphatic system clarifies the physiology of CNS metabolism and plays a vital role in the pathology of different neurological diseases, including neurodegenerative diseases, TBI, and stroke, serving as a promising target for intervention. However, most studies are limited to animal or cell experiments. More evidence is required to prove the similar effects of glymphatic pathway in humans. Future research on the glymphatic pathway must demonstrate its pathological change in human diseases and provide novel therapies.

## Figures and Tables

**Figure 1:** The glymphatic system functions as an interchange between cerebrospinal fluid (CSF) and interstitial fluid (ISF) and facilitates their exchange to promote waste removal. CSF within the subarachnoid space flows into the parenchyma via the periarterial space and subsequently exchanges with ISF, which is facilitated by astrocytic aquaporin-4 and drives the convective flow of interstitial solutes and ISF into perivenous spaces. Eventually, mixed CSF, ISF, and interstitial solutes flow along the perivenous space to remove metabolic waste products away from the brain parenchyma.

**Figure 2:** Schematic diagram of the circulation of cerebrospinal fluid (CSF) in the brain. CSF secreted by the choroid plexus flows into the subarachnoid space through the apertures of Magendie and Luschka of the fourth ventricle and then enters the perivascular spaces (glymphatic system). CSF collected alongside perivascular spaces ultimately drains into the periphery through meningeal lymphatics, arachnoid villi, the cribriform plate, and the spinal nerve root.

**Table 1:** Recently published human studies on the glymphatic system and meningeal lymphatics.

References	Year	Subjects or samples (list only human)	Imaging and mapping techniques	Main findings
Absinta et al. [16]	2017	5 healthy volunteers (three women, age range 28–53 years) and 3 healthy adult common marmosets (one female, two males, age range 4–11 years)	T2-FLAIR and T1-weighted black-blood MRI imaging, with gadolinium-based contrast agents	The existence of lymphatic vessels within the dura mater of human and nonhuman primates
Louveau et al. [17]	2015	9 autopsy specimens of human dura including the superior sagittal sinus	Leica TCS SP8 confocal system, Lyve-1 staining	The lymphatic structures were identified in two of nine human samples
Zhou et al. [52]	2020	35 patients (18 males, mean age: 52 years, age range: 21–71 years; 17 females, mean age: 58 years, age range: 18–79 years) with neurological disorders	Head T1-weighted imaging and head high-resolution T2-FLAIR MRI imaging, with contrast agent: gadodiamide	Glymphatic pathway and pMLVs might be impaired in the aging human brain; pMLVs are the downstream of the glymphatic pathway
Hasan-Olive et al. [59]	2019	Cortical brain biopsies of 30 iNPH patients (15 males and 15 females, mean age: 71 years) and 12 reference patients (6 males and 6 females, mean age: 44 years)	Semiquantitative immunogold electron microscopy	Perivascular AQP4 expression was attenuated in iNPH patients, potentially contributing to impaired glymphatic clearance
Kiviniemi et al. [62]	2016	9 healthy volunteers (5 females, age range: 21–30 years)	Novel multimodal ultrafast MREG technology	Three distinct pulsation mechanisms of the human glymphatic system coexist, and these pulsations can be separated using ultrafast MRI techniques

FLAIR: fluid-attenuation inversion recovery; MRI: magnetic resonance imaging; pMLVs: putative meningeal lymphatic vessels; iNPH: idiopathic normal pressure hydrocephalus; AQP4: aquaporin-4; MREG: magnetic resonance encephalography.

## Data Availability

No data were used to support this study.

## Abbreviations

A*β*: Amyloid *β*
AD: Alzheimer's disease
ApoE: Apolipoprotein E
AQP: Aquaporin
BBB: Blood-brain barrier
CAA: Amyloid angiopathy
COVID-19: Novel coronavirus- (SARS-CoV-2-) infected disease
CNS: Central nervous system
CSF: Cerebrospinal fluid
CTE: Chronic traumatic encephalopathy
DAPC: Dystrophin-associated protein complex
DCI: Delayed cerebral ischemia
dCLNs: Deep cervical lymph nodes
ePVS: Enlarged perivascular space
FTD: Frontal-temporal dementia
GFAP: Glial fibrillary acidic protein
ICH: Subarachnoid hemorrhage
ICP: Intracranial pressure
ISF: Interstitial fluid
MCAO: Middle cerebral artery occlusion
MRI: Magnetic resonance imaging
mTBI: Mild traumatic brain injury
NFT: Neurofibrillary tangle
NMDA: N-Methyl-D-aspartate acid
PUFAs: Polyunsaturated fatty acids
SAH: Subarachnoid hemorrhage
SAS: Subarachnoid space
sCLNs: Superficial cervical lymph nodes
SMC: Smooth muscle cell
TBI: Traumatic brain injury.
